The article "Neonatal NMDA Receptor Blockade Disrupts Spike Timing and Glutamatergic Synapses in Fast Spiking Interneurons in a NMDA Receptor Hypofunction Model of Schizophrenia" was published in 2014. Journal: PLoS One.

# Neonatal NMDA Receptor Blockade Disrupts Spike Timing and Glutamatergic Synapses in Fast Spiking Interneurons in a NMDA Receptor Hypofunction Model of Schizophrenia

**DOI:** 10.1371/journal.pone.0109303

**Published:** 2014-10-07

**Authors:** Kevin S. Jones, Joshua G. Corbin, Molly M. Huntsman

**Affiliations:** 1 Biology Department, Howard University, Washington, DC, United States of America; 2 Center for Neuroscience Research, Children’s National Medical Center, Washington, DC, United States of America; 3 Department of Pharmaceutical Sciences, Skaggs School of Pharmacy and Pharmaceutical Sciences, and Department of Pediatrics, School of Medicine, University of Colorado, Anschutz Medical Campus, Aurora, CO, United States of America; Chiba University Center for Forensic Mental Health, Japan

## Abstract

The dysfunction of parvalbumin-positive, fast-spiking interneurons (FSI) is considered a primary contributor to the pathophysiology of schizophrenia (SZ), but deficits in FSI physiology have not been explicitly characterized. We show for the first time, that a widely-employed model of schizophrenia minimizes first spike latency and increases GluN2B-mediated current in neocortical FSIs. The reduction in FSI first-spike latency coincides with reduced expression of the Kv1.1 potassium channel subunit which provides a biophysical explanation for the abnormal spiking behavior. Similarly, the increase in NMDA current coincides with enhanced expression of the GluN2B NMDA receptor subunit, specifically in FSIs. In this study mice were treated with the NMDA receptor antagonist, MK-801, during the first week of life. During adolescence, we detected reduced spike latency and increased GluN2B-mediated NMDA current in FSIs, which suggests transient disruption of NMDA signaling during neonatal development exerts lasting changes in the cellular and synaptic physiology of neocortical FSIs. Overall, we propose these physiological disturbances represent a general impairment to the physiological maturation of FSIs which may contribute to schizophrenia-like behaviors produced by this model.

## Introduction

Deficits to inhibitory neurotransmission are highly implicated in the etiology of schizophrenia (SZ) [1], as immunohistochemical analyses of post-mortem brain tissue often reveal decreases in the expression of one or more biochemical markers for gamma-aminobutyric acid (GABA) signaling [1]. Expression of the calcium binding protein, parvalbumin (PV), is particularly diminished in the neocortex of many SZ patients [2], which implies dysfunction of PV-expressing interneurons [3]. PV-expressing interneurons are physiologically distinguished by their capacity to discharge action potentials (“spikes”) at very high frequency and are thus termed “fast spiking” interneurons [4]. FSIs are interconnected via chemical and electrical synapses [5]–[7] which helps synchronize their own firing patterns [8], [9], and pace the firing patterns of large networks of pyramidal cells [10]. FSIs are thus integral for generating neural oscillations [11], [12], which incidentally, are often compromised in SZ patients. Although FSI dysfunction is highly inferred in the pathophysiology of SZ [13], physiological support for this hypothesis is lacking, particularly at the single cell level.

The NMDA receptor hypofunction model of SZ is founded on the discovery that acute administration of non-competitive NMDA antagonist (e.g. PCP, ketamine, and MK-801) evokes behaviors in healthy humans that are highly reminiscent of psychosis in SZ patients [14] [15]. Moreover, these drugs elicit behavioral deficits in animal models that closely model aspects of SZ [16]; [17] and also replicate disruptions in GABAergic biochemical markers. Administration of non-competitive NMDA receptor antagonist during early development is a particularly robust approach to model SZ-like biochemical deficits to GABA signaling [18]–[23]. Electrophysiological characterization of the NMDA hypofunction model of SZ has recently begun [24], but remains incomplete. Since direct physiological evaluation of FSIs in SZ patients is unfeasible, electrophysiological characterization of FSIs in animal models of SZ may be an expedient approach to identify specific impairments in FSI function.

In this study neonatal mice were treated with the NMDA receptor antagonist, MK-801, on postnatal day (PND) 6–8. The impact of neonatal MK-801 treatment on FSI physiology was then assessed during adolescence. This approach allowed us to directly test the hypothesis that transient disruption of NMDA receptor activity during early development causes persistent impairments to the function of neocortical FSIs. Whole-cell patch-clamp electrophysiology revealed that neonatal MK-801 treatment dramatically altered the spiking kinetics and action potential dynamics of FSIs. Pharmacological analysis revealed an increase in GluN2B-mediated NMDA current at excitatory synapses of FSIs from MK-801-treated mice. Immunohistochemical analyses identified congruent changes in the expression of key ion channel subunits that corroborate both sets of physiological data.

## Methods and Materials

### Experimental Animals

#### Ethics Statement

All animal use procedures were carried out in strict accordance with National Institutes of Health Guide for the Care and Use of Laboratory Animals and were approved by the Institutional Animal Care and Use Committee at Children’s National Medical Center.

To aid visualization of FSIs, we utilized transgenic mice that expressed the fluorescent reporter, Enhanced Yellow Fluorescent Protein (EYFP), exclusively in PV^+^ interneurons. These *PV-Cre^+/−^; Rosa26EYFP^loxP+^* mice were obtained by crossing a transgenic strain expressing cre recombinase under the control of the endogenous parvalbumin promoter (*PV-cre*); and a strain expressing a loxP-flanked *Rosa26-EYFP* marker (Jackson Laboratories, Maine). Only male mice were used in this study as sexually dimorphic responses to MK-801 have been reported [25], [26]. Male mouse pups were randomly assigned to the control or experimental group on PND6 and administered a subcutaneous injection of 0.75 mg/kg MK-801 (Tocris, USA) or an equal volume of saline for three consecutive days.

### Preparation of Brain Slices for Electrophysiology

Three to six week-old mice were anesthetized by carbon dioxide exposure and decapitated (*N* = 9, from 4 litters (vehicle-treated); *N* = 13, from 5 litters (MK-801-treated). Brains were rapidly removed to ice-cold, oxygenated (95% O_2_/5% CO_2_) sucrose-based slicing solution (in mM): 234 sucrose, 11 glucose, 24 NaHCO_3_, 2.5 KCl, 1.25 NaH_2_PO_4_*H_2_O, 10 MgSO_4_ and 0.5 CaCl_2_. Brains were trimmed, glued to a stage, and immersed in cold slicing solution. The somatosensory cortex (S1) was cut into 300 uM thick coronal slices with a vibrating microtome (Leica 1200S, Germany) and transferred to an incubation chamber containing oxygen-saturated artificial cerebral spinal fluid (aCSF) comprised of (in mM): 126 NaCl, 26 NaHCO_3_, 10 glucose, 2.5 KCl, 1.25 NaH_2_PO_4_*H_2_O, 2 MgCl_2_*6H_2_O, and 2 CaCl_2_*2H_2_O; pH 7.4. Modified coronal slices were used in a subset of experiments to retain a complete thalamocortical circuit [27], [28]. Slices were incubated at 32°C for one hour, then placed at ambient temperature (21–23°C) for 30 minutes prior to recording. Brain slices were placed into a recording chamber and visualized with a fixed staged, upright microscope (Nikon, FN1) equipped with 4x and 60x objectives, fluorescent filters, infrared (IR) illumination, Nomarski optics, and an IR-sensitive video camera (Cool Snap EZ, Photometrics).

### Electrophysiological recordings

Whole-cell patch-clamp recordings of FSIs were obtained under continuous perfusion of oxygenated aCSF (∼2 ml/min). Non-filamented glass pipettes (King Precision Glass, USA) were pulled on a vertical puller (PC-10, Narishige) to obtain electrodes with resistances of 3–5 MΩ when filled with an intracellular solution (in mM): 70 KCl, 70 potassium gluconate, 10 HEPES, 10 EGTA, 2 MgCl_2_, 4 Mg-ATP, 0.3 Na-GTP. Spontaneous excitatory and inhibitory events were acquired using a cesium-based intracellular solution comprised of (in mM): 20 KCl, 100 cessium methanesulfonate, 10 HEPES, 4 Mg-ATP, 0.3 Na-GTP, 3 QX-314 [29].

A GΩ seal was formed between the cell and glass pipette and a solenoid-controlled vacuum transducer was used to apply brief suction pulses (120 psi at 20–50 ms) to break into the cell. Recordings were acquired with pClamp 10 and a MultiClamp 700B amplifier (Molecular Devices, Sunnyvale, CA). Capacitance and series resistance compensation were used (typically 80%), and series resistance was continuously monitored throughout experiments. Putative FSIs were visually identified by EYFP fluorescence and then biophysical responses to brief hyperpolarizing and depolarizing current injections were characterized to confirm identity. The rheobase current (Ith) was determined as the minimum current amplitude capable of discharging a single spike for three consecutive trials. To accurately measure Ith, the amplitude of injected current was incrementally increased by 1–5 pA per sweep. Most cells discharged a single spike at Ith, (9/10 cells recorded in 10 slices from 9 vehicle-treated animals; 13/17 cells recorded in 17 slices from 13 MK-801-treated animals). Any cell which did not discharge a single spike was omitted from the study. Phase plots were constructed by calculating the first derivative (dV/dt) of I_th_ and plotting the value versus membrane potential (*Vm*).

For evoked recordings, depolarizing current pulses were delivered once every 15 seconds (Isoflex, A.M.P.I.; CPI, Carl Pisaturo, Stanford University). A minimal stimulation protocol was used to evoke EPSCs with a failure rate of approximately 50%. The amplitude of the current pulse ranged from 8.8–150 µA, with a fixed duration of 0.2 ms. EPSCs were evoked at the thalamocortical synapses of layer IV FSIs by placing a 25 µm concentric bipolar microelectrode (FHC, Bowdoin, ME) directly in contact with fibers projecting from the ventrobasal complex of the thalamus. EPSC amplitude was measured from the baseline to the peak of the initial response. The averaged EPSC decay time was fit to the double exponential function: *ƒ(t) = A_1_exp^−t/^*τ*^1^+A_2_exp^−t/^*τ*^2^*. These fits were used to determine a weighted time constant: τ_W_ = (τ_1_α_1_+τ_2_α_2_)/(α_1_+α_2_) where α and τ is the amplitude and time constant, respectively. NMDA currents were pharmacologically isolated by adding 20 uM glycine (Sigma), 20 uM 6,7-Dinitroquinoxaline-2,3-dione (DNQX, Tocris) and 10 uM SR 95531 hydrobromide (Gabazine, Tocris) to the perfusate.

### Analysis of Electrophysiology Data

Electrophysiological analyses were performed offline using Clampfit v10.2 (Molecular Devices, Sunnyvale CA) and Mini Analysis Program (Syanptosoft, Decatur, GA).

### Immunohistochemistry

Mice were anesthetized with isoflurane. An incision was made into the thoracic cavity, the rib cage was removed and mice were transcardially perfused with 20 mL of ice cold phosphate buffered saline (PBS) followed by 20 mL of an ice cold 4% paraformaldehyde (PFA) solution. The brain was removed and fixed overnight in 4% PFA. Brains were immersed in agar and cut into coronal sections (50 uM). Primary antibody staining was performed by incubating free-floating sections in a solution of PBST (PBS+0.2% Tween) +10% normal goat serum with the one or more of the following antibodies: mouse, anti-parvalbumin (Sigma, St. Louis, MO); goat, anti-NR2B (Abcam, Cambridge, MA); rabbit anti-parvalbumin (Savant, Switzerland); and mouse Kv1.1 (UC Davis/NIH NeuroMab Facility). Sections were shaken overnight at 4°C, then washed five times in PBST and incubated overnight at 4°C in a solution of PBST+10% normal donkey serum and the following secondary antibodies: donkey, anti-rabbit Alexa 488 (Invitrogen); donkey, anti-mouse Alexa 555 or donkey anti-goat Alexa 555. Sections were washed, mounted, and covered with a glass cover slip. Confocal micrographs were captured on a Leica LSM 510 confocal microscope equipped with 10x, 20x, 40x oil, 63x oil, and 100x oil objectives. Post-hoc immunohistochemical analysis confirmed all fluorescently labeled cells were positive for parvalbumin.

### Statistical Analysis

Data are expressed as mean +/− SEM. Differences among experimental groups were considered statistically significant at *p*<.05. ANOVA and two-tailed, Student’s T-Test was used to compare changes between each experimental group.

## Results

### Neonatal NMDA Receptor Blockade Minimizes First-Spike Latency in Neocortical FSIs

The electrophysiological development of FSIs in the mouse somatosensory cortex (S1) has been comprehensively characterized [30], and FSIs from S1 may also be highly vulnerable to perinatal NMDA receptor blockade [18]. We therefore chose FSIs from S1 as the subject of this study to maximize sensitivity to MK-801 treatment.

The onset of action potential discharge (or “spiking”) varies widely in neocortical FSIs and is inversely proportional to stimulus strength [31]. Strong stimuli elicit spikes from FSIs rapidly, whereas near-threshold level stimuli elicit spikes with a temporal delay, termed first-spike latency [31]. We found that first-spike latency was significantly shorter in FSIs from MK-801-treated mice compared to vehicle-treated mice [MK-801-treated: 12.5±1.7 ms (SEM), *n* = 11 cells; *versus* Vehicle-treated: 43.8±17.0 ms, *n* = 9 cells; *P* = 0.02] (Figures 1A, B). Since first-spike latency is inversely proportional to stimulus intensity, we examined the relation of stimulus intensity to first-spike latency to more closely assess the impact of neonatal MK-801 treatment on the input-output function of FSIs. A log-log plot confirmed first-spike latency is, indeed, inversely proportional to stimulus intensity when spikes are discharged by low-to-moderate strength stimuli (e.g. current amplitude of <2x I_th_) (Figure 1D). However, when spikes were discharged by high intensity stimuli (e.g. >2x of I_th_), the relation of stimulus intensity to first-spike latency became non-linear and a stable, stimulus-insensitive function appeared in FSIs from saline-treated mice (Figure 1D). By contrast, first-spike latency in FSIs from MK-801 treated mice remained inversely proportional at all stimulus intensities (Figure 1E). This permitted spikes with substantially shorter latencies to be discharged by high intensity stimulation. These data suggest first-spike latency is comprised of at least two components in FSIs which exhibit distinct relationships to stimulus intensity. Moreover, neonatal NMDA receptor blockade appears to shorten the stimulus-insensitive component of first-spike latency.

**Figure 1:** Postnatal NMDA receptor blockade decreases first-spike latency in neocortical layer IV FSIs. (A, B) Prototypical discharge patterns of FSIs from a vehicle- or MK-801-treated mouse. Traces show voltage response to 600 ms injections of current at saturating (black trace), or threshold (red trace) amplitude. Red arrows below trace indicate onset of current injection and spike threshold (defined as dVm/dt>10). Solid red bar below trace illustrates delay to first spike (C) Quantification of delay to first spike at rheobase response. Values are means ± S.E.M. *P<0.05, vs. control. (D, E). A log-log plot of first spike delay versus amplitude of injected current in layer IV FSIs from vehicle- (D) or MK-801–treated mice (E). Dashed lines on the y-axes illustrate spike latency of log 0.3 ms (or 2.0 ms log_10_).

### Neonatal NMDA Receptor Blockade Alters Several Intrinsic Spiking Properties of Neocortical FSIs

Many intrinsic properties of FSIs are optimized to deliver precisely timed spikes [32] that exhibit very little frequency accommodation during spike trains [4]. For instance, FSIs exhibit a low input resistance, fast membrane time constant, and narrow spike width [33]. All of these attributes help FSIs discharge spikes with high temporal precision and at a sustained rate. We characterized several active and passive membrane properties of FSIs to determine the impact of neonatal MK-801 treatment. The input resistance of FSIs from MK-801 treated mice was 50.3% higher than vehicle-treated mice [Rin; MK-801-treated: 154.8±13.4 MΩ (SEM), *n* = 13; Vehicle-treated: 103.0±8.1 MΩ. *n* = 9; *P*<0.01, Table 1]. Spikes discharged from the FSIs of MK-801-treated mice were 14.6% broader than vehicle-treated mice [AP ½ width: MK-801-treated: 0.47±0.01 ms (SEM), *n* = 13; Vehicle-treated: 0.41±0.02 ms, *n* = 9; *P*<0.01, Table 1] and displayed significantly more spike frequency accommodation [spike frequency accommodation ratio: MK-801-treated: 0.73±0.02 ms (SEM), *n* = 13; Vehicle-treated: 0.94±0.10 ms, *n* = 9; *P*<0.05, Table 1]. The maximum firing rate of FSIs from MK-801-treated mice was 17% lower than FSIs from vehicle-treated mice, although this difference was not statistically significant (*P = *0.11). Together these data suggest neonatal NMDA receptor blockade disrupts both active and passive membrane properties of neocortical FSIs which could subsequently impair spiking behavior.

**Table 1:** Electrical properties of layer IV FS neurons in the Somatosensory Cortex.

	Vehicle-Treated	MK-801-Treated
**Passive Intrinisic Properties**		
R_in_ (MΩ)	**103.0±8.1 (9)**	**154.8±13.4** ** **(13)**
V_rest_ (mV)	−65.5±1.8 (9)	−66.9±1.1 (13)
τ_m_ (ms)	6.8±0.8 (9)	8.5±0.8 (11)
I_h_ (mV)	4.00±0.5 (7)	3.75±0.9 (7)
**Active Intrinsic Properties**		
I_th_ (pA)	190±45 (9)	140±20 (13)
Max. Spike Freq. (Hz)	161.8±9.9 (9)	138.7±16.9 (9)
AP half-width (ms)	**0.41±0.02 (9)**	**0.47±0.01** ** **(13)**
AP accommodation ratio	**0.94±0.10 (9)**	**0.73±0.02** * **(13)**
AP threshold (mV)	−41.9±3.2 (9)	−34.0±6.5 (13)
AHP Amplitude (mV)	17.1±2.5 (9)	15.5±1.3 (13)
Ratio 1st/2nd AHP Amp.	1.02±0.01 (9)	1.01±0.003 (13)
t_AHP peak_ (ms)	3.41±0.08 (9)	3.63±0.34 (12)

*P<0.05;

**P<0.01.

*V*rest, resting membrane potential; *R*_in_, input resistance; τ_m_, membrane time constant. Data are mean ± SEM. Numbers in parantheses are *N.*Selected values shown in bold are significantly different from the same parameter measured in control cells.

*Value is significantly (*P*<0.05) different from control.

**Value is significantly (*P*<0.01) different from control.

Resting membrane potential (Vrest) was recorded within the first two minutes after break in. Input resistance (Rin) was calculated from the voltage response measured at the end of hyperpolarizing current steps (600 ms). Membrane time constant (τ) was obtained by fitting a single exponential to the relaxation of membrane potential (Vm) to a −300 pA current injection. Ih current was calculated by the formula Vm2−Vm1, where Vm2 was measured at the end of a −300 pA current step and Vm1 was measured at the maximal hyperpolarization. Depolarizing currents were injected to elicit action potentials (AP) and the AP firing patterns were used to characterize accommodation ratio, APl duration at half-width, AP amplitude and rise time. Single AP properties were measured from the first AP elicited by a minimally supra-threshold current step which elicited a continuous train of APs. AP firing threshold was determined by differentiating the voltage trace (dV/dt) evoked by the current step in current-clamp mode. The voltage and time at which the first AP discharged were taken as the value at which dV/dt≥10. In all recordings, this value exceeded baseline values (an average of the preceding 10–100 ms) by≥20-fold. AP half-width was defined as the period between the half-amplitude point in the rising and decaying phase of the AP. The ratio of the 1st AP/2nd AP was calculated using the peak amplitudes as one measure of accommodation. The ratio of the interval between the first APs and the average interval of the last three APs during a train was calculated as a second measure of AP accommodation. The after hyperpolarization (AHP) amplitude was calculated as the difference from AP threshold to the maximum trough of hyperpolarization.

### Neonatal NMDA Receptor Blockade Destabilizes Spike Threshold Dynamics

The spike threshold of layer IV neocortical neurons can be dynamic [34]. We characterized the spike threshold dynamics of neocortical FSIs to assess the impact of neonatal NMDA receptor blockade. We first examined spike threshold at I_th_. I_th_ was determined, as previously described, and phase plots were constructed for each cell to allow spike threshold to be determined graphically (Figure 2). Spike threshold at I_th_ was about 8 mv more depolarized in FSIs from MK-801-treated mice, although this difference was not statistically significant [Vehicle-treated: −41.9±3.2, *n* = 9 versus MK-801-treated: −34.0±6.5 mV, *n* = 13; *P* = 0.34, Table 1]. The amplitude of the I_th_ current was incrementally increased in successive sweeps to examine the dynamics of spike threshold (Figure 2C–F). The spike threshold of FSIs from vehicle-treated mice was examined across a broad range of stimulus intensities and found to be stable and independent of current amplitude (Figure 2G). By contrast, FSIs from MK-801-treated mice exhibited a positive correlation to current amplitude [slope in MK-801-treated FSIs: 0.018±0.004 pA mV^−1^, *n* = 8; versus slope of vehicle-treated FSIs: −0.004±0.004 pA mV^−1^, *n* = 8; *P* = 0.003] (Figure 2I). These data suggest stimulus intensity has a larger influence on the spike threshold of FSIs from MK-801-treated mice, and that the dynamics of spike threshold are also less stable than in FSIs from vehicle-treated mice.

**Figure 2:** Postnatal NMDA receptor blockade destabilizes spike threshold in neocortical layer IV FSIs. (A, B) Representative voltage responses of first spikes elicited from FSIs at rheobase (I_th_); I_th_+100 pA; I_th_+200; and I_th_+300 pA current steps. For clarity, only the initial spike in each trace is displayed, and the intervening, +50 pA, current steps are omitted. (C, D) Phase plots of the traces shown in A, B. Phase plots are shown for the first spike discharged during injection at I_th_ and I_th_ +: 50, 100, 150, 200, 250 and 300 pA. (E, F) Regions of interest indicated by the dashed line are displayed at higher magnification. Red dashed line indicates spike threshold (dV/dt = 10). Insets are plots of injected current amplitude versus first spike threshold of displayed cell. (G, H) Plots of injected current amplitude versus first spike threshold. (I) Mean slope of injected current amplitude versus first spike threshold in (G, H). Values are means ± S.E.M. **P<0.005, vs. control by ANOVA.

### Neonatal NMDA Receptor Blockade Reduces Kv1.1 Expression in Neocortical FSIs

Both first-spike latency and spike threshold are strongly modulated by K^+^ channels comprised from Kv1 potassium channel subunits [34]. In neocortical FSIs, first-spike latency is specifically mediated by the Kv1.1 subunit [31]. We therefore hypothesized the alterations in first-spike latency and spike threshold dynamics observed in FSIs from MK-801-treated mice resulted from disturbances in the expression of the Kv1.1 subunit. Immunohistochemical analysis revealed that neonatal MK-801 treatment dramatically reduced staining for the Kv1.1 subunit in neocortical FSIs (Figures 3A–H). These findings are consistent with our physiological characterizations and demonstrate that transient, NMDA receptor blockade during early development can reduce expression of the Kv1.1 subunit in the FSIs of adolescent mice.

**Figure 3:** Postnatal NMDA receptor blockade reduces somatic expression of Kv1.1. (A–H) Representative confocal micrographs (maximal intensity, flattened Z-stack, z separation of 1.03 um) of somatosensory cortex from adolescent mice (PND42) neonatally injected with vehicle (A–D), or MK-801 (E–H). (D, H) Staining for the Kv1.1 potassium channel subunit is dramatically reduced in FSIs from MK-801-injected mice. Insets in (B) and (F) show higher magnification of layer IV regions of interest. Green = Parvalbumin; Red = Kv1.1. Scale bars = 100 um (A–C; E–G) or 10 um (D, H and insets in B, F).

### Neonatal NMDA Receptor Blockade Increases Mg^2+^-Sensitive sEPSCs onto FSIs

We next evaluated the impact of neonatal NMDA receptor blockade on synaptic input to FSIs. Whole-cell patch clamp recordings from neocortical FSIs revealed the average frequency of sEPSCs recorded from FSIs of MK-801-treated mice was 50% higher than vehicle-treated mice, although statistical significance was not reached [Vehicle-treated: 21.2±4.4 Hz, *n* = 6; *versus* MK-801-treated: 31.4±2.7, *n* = 8; *P* = 0.06] (Figure 4A). NMDA-mediated EPSCs may be highly sensitive to Mg^2+^ block [35], [36], so we repeated these experiments in superfusate with 0 mM added Mg^2+^ (Figures 4A, B). In nominal Mg^+^, the frequency of sEPSCs recorded from the FSIs of MK-801-treated mice was 60% higher than sEPSCs recorded from vehicle-treated mice and statistically significant [Vehicle-treated: 16.1±2.51 Hz, *n* = 4; *versus* MK-Treated: 26.1±2.21 Hz, *n* = 8; *P* = 0.03] (Figure 4B). There was no difference in sIPSC frequency at either concentration of Mg^2+^ (Figure 4B), thus inhibitory currents were not examined further.

**Figure 4:** Postnatal NMDA receptor blockade increases glutamatergic input to neocortical FSIs. (A) Representative whole-cell patch clamp recordings from FSIs in acute brain slices from the somatosensory cortex of adolescent mice (PND21-P25) neonatally-treated with vehicle or MK-801. Spontaneous activity was recorded in 2 mM (left traces) or 0 mM (right traces) of added Mg^2+^. Recordings were obtained in voltage clamp mode. sIPSCs (top traces) were recorded at the sEPSC reversal potential (∼+10 mV) and sEPSCs (bottom traces) were recorded at the Cl- reversal potential (∼−40 mV). (B) Bar graphs of mean sEPSCs and sIPSCs frequency obtained during 5 min recordings. Values are means ± S.E.M. *P<0.05, vs. control by ANOVA.

### Neonatal NMDA Receptor Blockade Increases NMDA Current at the Thalamocortical Synapses of FSIs

The increase in sEPSC frequency that occurs in 0 mM Mg^2+^ superfusate could result from increased NMDA-mediated events or increased α-amino-3-hydroxy-5-methyl-4-isoxazolepropionic acid (AMPA)-mediated events. Moreover, since layer IV FSIs receive excitatory input from both thalamocortical circuits [28], [37] and local layer IV spiny stellate cells [38] the origin of the Mg^2+^-sensitive sEPSCs was not clear. To more clearly distinguish the source of the Mg^2+^-sensitive sEPSCs we utilized a thalamocortical slice preparation. In this preparation, monosynaptic AMPA currents were evoked onto FSIs from vehicle-treated or MK-801-treated mice (V_HOLD_ = −60 mV). The average amplitude of AMPA current was similar between the two groups [Vehicle-treated: 97.2±13.0 pA, *n* = 3; MK-801-treated: 87.3±23.6 pA, *n* = 3; *P* = 0.36] (Figures 5A, D), and no difference was detected in the 10–90% rise time [Vehicle-treated: 1.8±0.1 ms, *n = *3; MK-801-treated: 2.1±0.7 ms, *n = *3; *P* = 0.32] or decay time [Vehicle-treated: 3.0±1.2 ms, *n = *3; MK-801-treated: 4.8±1.3 ms, *n = *3; *P* = 0.18] of evoked AMPA current (Figures 5B, C, E, F).

**Figure 5:** Postnatal NMDA receptor blockade increases expression of functional NR2B receptors in neocortical FSIs. Prototypical excitatory post-synaptic currents were evoked onto layer IV FSIs in a thalamocortical slice preparation. (A–C) AMPA-mediated responses were similar in vehicle-treated mice (black traces) and MK-801-treated mice (red traces). (V_Hold-AMPA_ = −60 mV). Traces shown are the average of 5–10 responses obtained at the same stimulus intensity from vehicle-treated mouse (black lines); or MK-801-treated mouse (red lines). Dashed boxes designate regions of interest in activation and decay kinetics. (D–F) Bar graphs of mean current amplitude and mean weighted activation tau (τ_w_Act.) and deactivation tau (τ_w_Deact.) of evoked AMPA current evoked from vehicle-treated mice (black bars) and MK-801-treated mice (red bars). (G, H) The kinetics of NMDA-mediated responses are slower in MK-801-treated mice (red traces). (V_Hold-NMDA_ = +60 mV). Traces shown are the average of 5–10 responses obtained at the same stimulus intensity. Dashed boxes designate regions of interest in activation and decay kinetics. (I–K) Bar graphs of mean current amplitude and mean weighted activation tau (τ_w_) and deactivation tau (τ_w_) of evoked NMDA current from vehicle and MK-801-treated mice. Values are means ± S.E.M. *P<0.05, vs. control by ANOVA. (L–S) Representative confocal micrographs of layer IV somatosensory cortex from mice neonatally treated with vehicle (L–O), or MK-801 (P–S). (L, P) Dashed boxes designate regions of interest in layer IV selected for higher magnification as shown in (M–O), and (Q–S). Green = Parvalbumin; Red = GluN2B. Scale bars = 100 um (L, P) or 10 um (M–O; Q–S). Images are shown as a maximum intensity projection of single images at a Z-spacing of 1.0 uM. (N, R) Arrowheads denote GluN2B staining as puncta or broad staining in brain slices from a vehicle-treated, or MK-801-treated mouse, respectively. (T–W) Representative traces of ifenprodil blockade on monosynaptic NMDA current evoked onto a FSI from an adolescent mouse neonatally treated with vehicle (T) or MK-801 (V) Traces shown are averages of 5–10 responses to the same stimulus intensity before (black lines) and after (grey lines) 10 minute wash in of 3 uM Ifenprodil. (U, W) Same traces as shown in (T) and (V) scaled on y-axis to facilitate visual comparison of the actions of ifenprodil on activation and decay kinetics. Average traces were fit, as previously described. (X, Y, Z) Quantitative analysis of impact of ifenprodil on mean peak amplitude (X); mean reduction in total charge (Y); and mean change in τ_w_ decay (Z). (*N* = 4 cells from 4 animals (vehicle-treated); and 3 cells from 3 animals (MK-801-treated).

Although there was no difference in the peak amplitude of evoked NMDA current [Vehicle-treated: 131.4±105.5 pA, *n = 3*; MK-801-treated: 137.3±65.4 pA, n = 3; *P* = 0.49] (Figure 5G, I), both the 10–90% rise time and the decay time of evoked NMDA current was significantly slower in FSIs from MK-801-treated mice: [10–90% rise time: MK-801-treated: 37.9±12.4 ms, *n = 3*; Vehicle-treated: 5.2±1.7 ms, *n = *3; *P* = 0.02], [Average decay time: MK-801-treated: 170.4±9.7 ms, *n = 3*; Vehicle-treated: 54.3±12.0 ms, *n = 3, P* = 0.02] (Figures 5G, H, J, K). Together the increase in Mg^2+^-sensitive sEPSCs, and slower kinetics of the evoked NMDA current suggests neonatal NMDA receptor blockade alters the composition of NMDA receptors expressed at the thalamocortical synapses of layer IV FSIs.

NMDA receptors are comprised from heteromeric subunits [39] and the kinetic properties of the receptor channel are mostly determined by GluN2 subunits [40]. By adolescence, neocortical NMDA current is predominated by GluN2A and GluN2B-comprised receptors [41]. The GluN2B subunit confers slower channel kinetics to NMDA receptors [42], thus we hypothesized neonatal MK-801 exposure altered expression of GluN2B subunits in FSIs. Immunohistochemical analysis revealed neonatal MK-801 treatment increased GluN2B staining in FSIs (Figures 5R, S). The functionality of the surplus GluN2B subunits was examined by measuring the sensitivity of evoked NMDA current to the GluN2B-selective antagonist, ifenprodil [43]. Bath application of ifenprodil dramatically increased the decay rate of NMDA current evoked onto FSIs from MK-801-treated mice, but not vehicle-treated mice [% change τ_W_: Vehicle-treated, −9.9±13.7%, *n = *3; % change τ_W_: MK-801-treated, 55.6±4.0%, *n = 3*, *P* = 0.008] (Figures 5T, U, Z). Similarly, ifenprodil attenuated the peak amplitude and total charge of NMDA current evoked from MK-801-treated mice more strongly than vehicle-treated mice [% peak amplitude reduction *I*_NMDA_: Vehicle-treated, 49.5±1.7%, *n = *3; MK-801-treated, 80.4±2.4%, *n = 3*, *P* = 0.009] [% reduction *Q*_NMDA_: Vehicle-treated, 35.1±6.7%, *n = *3; MK-801-treated, 90.1±1.7%, *n = 3*; *P* = 0.009] (Figures 5X, Y). These data demonstrate neonatal MK-801 treatment substantially increased the proportion of GluN2B-mediated NMDA current at the thalamocortical synapses of layer IV FSIs.

## Discussion

Here we demonstrate that neonatal MK-801 treatment disrupts both intrinsic and synaptic functions of neocortical FSIs in adolescent mice. These findings support our hypothesis that transient neonatal NMDA receptor blockade causes persistent alterations in FSI physiology, and we now propose a mechanism by which these alterations could be mediated.

### Neonatal MK-801 Treatment May Minimize First-Spike Latency by Reducing Kv1.1 Expression in FSIs

Neonatal MK-801-treatment reduces expression of the Kv1.1 subunit (Figure 3) which we propose shortens first-spike latency in FSIs (Figure 1). First, consider that near resting membrane potential a substantial fraction of Kv1.1-comprised K^+^ channels are partially open [44]. Thus, during low amplitude stimulation a significant portion of the current injected during whole-cell patch clamp of FSIs leaks out as K^+^ ions (Figure 6A). This efflux of K^+^ ions slows the rate of membrane depolarization [45] [44] and delays spike discharge [44] (Figure 6B). Since neonatal MK-801 treatment reduces Kv1.1 expression (Figure 6C), the fraction of current that leaks during whole-cell patch clamp is minimized, increasing the rate of membrane depolarization, and minimizing first-spike latency (Figure 6D). This interpretation is further supported by the finding that the resting input resistance (R_in_) of FSIs from MK-801-treated mice is 50% higher than FSIs from vehicle-treated mice (Table 1) (*P*<0.01). Moreover, the amplitude of I_th_ in FSIs from MK-801-treated mice was smaller than vehicle-treated mice, although the difference did not reach statistical significance (Table 1). Together, these data support our interpretation that first-spike latency is shortened in FSIs from MK-801–treated mice because of reduced expression of the Kv1.1 subunit.

**Figure 6:** Schematic depiction of how neonatal MK-801 treatment impacts the spike timing of an FSI from an adolescent mouse. (A) A significant proportion of the current injected during whole-cell patch-clamp (yellow lightning bolts) dissipates through the high density of Kv1.1-containing K^+^ channels expressed in FSIs from vehicle-treated mice. (B) The time required to depolarize the cell membrane to threshold is increased and first-spike latency is temporally expanded. (C) By contrast, a lower proportion of injected current dissipates FSIs from MK-801-treated mice due to reduced expression of Kv1.1-containing K^+^ channels. (D) The time required to depolarize to threshold is reduced and first-spike latency is therefore minimized.

### Neonatal MK-801-treatment May Increase the Spike Threshold Dynamics of FSIs

Compared to FSIs from vehicle-treated mice, the spike threshold of FSIs from MK-801-treated mice is more dynamic and inversely correlated to stimulus intensity (Figure 2G, H). During periods of sustained or intense stimulation the spike threshold of FSIs from MK-801-treated mice could adapt to more depolarized values [46] and thereby reduce excitability. Interestingly, FSIs from MK-801-treated mice exhibit a reduced maximum spike rate and an increased spike accommodation ratio (Table 1). Increased spike-threshold dynamics may help explain these findings. It is not clear how neonatal MK-801 treatment might increase the spike-threshold dynamics of FSIs. However, K+ channels comprised from the Kv1.1 subunit have been shown to regulate spike-threshold variability [31], [34], [44]. Thus it is conceivable that the changes in FSI spike-threshold dynamics could result from changes in the expression and/or function of K+ channels comprised from the Kv1.1 subunit.

### Neonatal MK-801 Treatment May Impair Physiological Maturation of Neocortical FSIs

Our mechanistic model of how neonatal MK-801 treatment shortens first-spike latency was derived from a relatively straightforward interpretation of our results. However, a more expansive consideration of our findings supports the notion that neonatal MK-801 treatment may broadly impair physiological maturation of FSIs. Below we consider this idea within the context of our most salient findings–disrupted membrane properties, shortened first-spike latency, and increased GluN2B NMDA current.

The membrane properties and spiking characteristics of mature FSIs are highly specialized to facilitate the discharge of brief, precisely timed spikes. Specifically, spikes from mature FSIs exhibit a narrow spike width, low input resistance, fast membrane time constant, and low frequency accommodation ratio [47] [32] [33]. Curiously, these properties are not innately optimized, but rather undergo extensive refinement during the postnatal development of FSIs. For example, FSIs from immature mice have a high input resistance, slow membrane time constant, broad spike width and exhibit considerable spike frequency accommodation [33]. These immature features oppose the rapid and precise spiking activity that characterizes mature FSIs [47]. However, FSIs undergo rapid postnatal development, and by P18 they attain mature membrane properties and spiking characteristics that remain stable through adulthood [30].

In this study the membrane properties and spiking characteristics of FSIs were evaluated in adolescent mice aged adolescent mice aged PND 26±2.3. Notably, several of the membrane properties and spiking characteristics of FSIs from MK-801 treated mice were physiologically immature compared to FSIs from age-matched, vehicle-treated mice. For instance, the average membrane resistance and spike accommodation ratio of FSIs from MK-801-treated mice were significantly less mature than FSIs from vehicle-treated mice (Table 1). Similarly, the membrane time constant (τ_m_), steady-state firing rate, and instantaneous firing rate of FSIs from MK-801-treated mice were also less mature than FSIs from vehicle-treated mice (Table 1), though these differences did not reach statistical significance. Overall, the membrane properties and spiking characteristics of FSIs from MK-801-treated mice exhibited a level of physiological maturity comparable to FSIs from healthy mice aged ∼P13–15 [30]. We therefore conclude that transient, neonatal MK-801 treatment impairs biophysical maturation of neocortical FSIs. More broadly, these data suggest a role for NMDA signaling in the normal development of FSIs.

### Neonatal MK-801 Treatment May Impair Developmental Regulation of First-Spike Latency

FSIs can be distinguished by first-spike latency [48], but the development of this pattern has not been fully characterized. However, since first-spike latency is highly dependent on the Kv1.1 subunit (Goldberg et al 2008), it is likely to correlate with the developmental expression of the Kv1.1 subunit. In neonatal mice the expression of Kv1.1 mRNA is very low in neocortical FSIs, but the expression increases more than 40-fold by P21 [33]. If expression of the Kv1.1 subunit is monotonically regulated, first-spike latency in FSIs may progress with a similar developmental trajectory. If so, our finding that transient, neonatal MK-801 treatment reduces expression of the Kv1.1 subunit and shortens first-spike latency in the FISIs of adolescent mice further supports the notion that NMDA signaling contributes to the physiological development of neocortical FSIs.

### Neonatal MK-801 Treatment May Impair Maturation of Excitatory Synapses in Neocortical FSIs

The subunit composition of NMDA receptors is developmentally regulated. During early development, neocortical NMDA current is comprised mostly from GluN2B-containing receptors [49], [50]. During adolescence a stereotyped developmental switch occurs and the proportion of NMDA current mediated by GluN2B-containing receptors in FSIs diminishes [24]. Thus, the proportion of GluN2B-mediated NMDA current is approximately inversely proportional to FSI development. In this study NMDA current was characterized from the FSIs of adolescent mice (PND 42–45). Sensitivity to the GluN2B-specific antagonist, ifenprodil, was used to determine the contribution of GluN2B-mediated NMDA current. As expected, NMDA current evoked from the FSIs of vehicle-treated mice was comprised of only 35% GluN2B-mediated current, whereas NMDA current evoked from the FSIs of MK-801-treated mice was comprised of about 90% GluN2B-mediated current (Figures 5T–Z). While this study was in progress two reports emerged which corroborate our findings. In the first report, neonatal administration of a GluN2A-specific antagonist increased the proportion of GluN2B-mediated NMDA current evoked from FS cells in the somatosensory cortex of adolescent mice [24]. In the second report, perinatal administration of phencyclidine increased the expression of the GluN2B subunit in the prefrontal cortex of adolescent rats [51]. Together, these data suggest transient disruption of NMDA signaling may indelibly alter the ontogeny of excitatory synapses throughout the neocortex.

In summary, neonatal NMDA receptor blockade remains a robust approach for modeling many schizophrenia-like behavioral deficits in animals [17]. However, the pathophysiological mechanisms which give rise to the behavioral deficits are unclear. In this study we discovered that neonatal NMDA receptor blockade simultaneously *minimizes* first-spike latency and *increases* the proportion of GluN2B-mediated NMDA current at thalamocortical synapses onto neocortical FSIs. Both of these results are consistent with our general notion that neonatal MK-801 treatment impairs the physiological maturation of neocortical FSIs, and since layer IV FSIs process the majority of thalamic sensory input, it is conceivable that the disturbances in FSI physiology we report contribute to the pathophysiology underlying the schizophrenia-like behaviors.
